# Effect of Nursing Intervention in the Operating Room Based on Simple Virtual Reality Augmented Technology on Preventing Gastrointestinal Surgical Incision Infection

**DOI:** 10.1155/2021/9981821

**Published:** 2021-05-03

**Authors:** Yanhua Wang, Dan Zhang, Shujing Wei

**Affiliations:** ^1^Center Sterile Supply Department East Campus, Jining First People's Hospital, Jining 272000, Shandong, China; ^2^Operation Room, Jining First People's Hospital, Jining 272000, Shandong, China

## Abstract

Gastrointestinal surgery is currently a common gastrointestinal surgery in clinical practice. In recent years, the incidence of gastrointestinal diseases has gradually increased and increased as the lifestyle of modern people has developed and changed. Both physical health and quality of life have a serious impact. In the actual process, it was found that multiple links in operating room care may increase the risk of postoperative infections for patients. Therefore, this article proposes nursing in operating room based on simple virtual reality augmented technology. This article mainly studies the effect of nursing intervention on preventing gastrointestinal surgical incision infection, and hopes to provide help for preventing gastrointestinal surgical incision infection. In this trial, 80 patients with gastrointestinal surgery were randomly divided into two groups, each with 40 people. The experimental group was treated with an operating room nursing intervention combined with traditional treatment methods. Controls were treated with traditional nursing combined with traditional treatment, and both groups were analyzed for acceptance of nursing intervention in the operating room, poor mood, various indicator levels, postoperative complications, and postoperative incisional infections. The experiment proved that the postoperative rehabilitation indexes of the experimental group were better than those of the control group, the excellent rate of wound healing reached 92.5%, and the incidence of wound infection was only 5%, which was lower than that of the control group. This demonstrates that nursing intervention in the operating room can help to reduce the infection rate at the patient's incision site, increase the level of surgical indicators, promote healing of the incision site as quickly as possible, and significantly improve the safety of clinical treatment.

## 1. Introduction

Abdominal surgery is a common method of treatment of gastrointestinal diseases. This treatment method may cause various complications in patients after surgery. Common complications include incision pain, incision fever or redness, and varying degrees of infection in the affected area of the patient, which is perfect and the implementation of disinfection and isolation technology in the operating room is closely related to the occurrence of incision infection. If the patient does not receive proper disinfection and sterilization during surgery, the risk of exposure to bacterial infections increases significantly, which affects the effectiveness of surgical treatment and the patient's prognosis. Therefore, further studies on the effect of nursing interventions on the prevention of gastrointestinal infections caused by surgical incisions in the operating room are highly needed.

Research on the prevention of surgical wound infection in foreign countries is much faster than in China. At the same time, the application of operating room nursing intervention is faster than in China, and with the rapid development and update of operating room nursing intervention, intervention treatment methods and methods have become enormous. It is believed that in the near future the use of nursing intervention in the operating room will become an important breakthrough. In order to observe and analyze the impact of nursing intervention in orthopedic ward on incisional infection during aseptic surgery in orthopedic ward, Cooper selected patients and patients who underwent aseptic surgery, and reviewed why these patients and patients had incisional infection [1]. Endo comprehensively analyzed the clinical effects of operating room nursing intervention in preventing incision infection in patients undergoing gastrointestinal surgery and found that operating room nursing intervention is more ideal than conventional nursing mode [2]. Mubin believed that surgical incision infection will bring huge pain to patients, and more serious or even life-threatening, and proposed the operation room nursing intervention to prevent incision infection [3].

Treatment methods using operating room nursing interventions began in Western countries. Compared to Western countries, intervention treatment methods and methods in our country started late and their development is relatively slow. With the continuous development and development of modern science and technology and the increasing maturity of medical technology, the diagnosis and treatment level of gastrointestinal surgery in our country has improved, and the prognosis of patients has also improved. Zhang believes that it can enhance patients' positive attitude towards treatment and reduce anxiety, depression, and other negative emotions, so as to provide clinical reference for prolonging the survival time of cancer patients, improving the quality of life of patients and promoting the recovery of the disease [4]. Zhou proposed that patients with gastrointestinal malignant tumors who use operating room nursing intervention support during the operation period can promote postoperative recovery and reduce the occurrence of complications [5]. Liu analyzed the clinical data of 400 rectal cancer patients, and as a result of multivariate regression analysis, long-term hospitalization of rectal cancer patients after surgery was a predictor of postoperative chemotherapy delay [6].

In this paper, we study the effect of nursing intervention in the operating room on preventing gastrointestinal surgical incision infection, analyzing the patient's depression, anxiety, and other adverse emotional conditions, the patient's postoperative complications, and surgical incision infection, revealing that operating room nursing intervention is effective in preventing stomach infections. OTC incision infections play a role in reducing the likelihood of gastrointestinal incision infections, leading to widespread promotion of operating room nursing interventions in gastrointestinal surgery clinics, providing new information for more in-depth research into the application of operating room nursing interventions.

## 2. Effect of Nursing Intervention on Preventing Gastrointestinal Operative Incision Infection

### 2.1. Process of Virtual Reality Augmented Vision to Generate Pictures

The purpose of image preprocessing is to ensure the accuracy of the next image input, make some folding changes, and coordinate transformations in the original image, or capture and enhance the image of a noisy image. It mainly includes basic image editing functions, image mapping templates, image conversion, and export image feature sets, etc., pre-positioning, finding approximate overlapping areas, reducing the mapping range, and increasing speed.

#### 2.1.1. Transformation Model

During the image capture process, the state of the image is determined by the movement of the camera. In general, camera movement can be divided into parallel movement, lens zoom, horizontal scan, vertical scan, and rotation movement [7, 8]. Different ways of moving the camera will produce different effects in the scene. The complex movement of the camera will inevitably make different image sequences in space, especially overlapping image sequences. Due to the complex movement of the camera, a large number of coordinate transformations before the image are required, including rigid body transformation, correlation transformation, and projection transformation.

#### 2.1.2. Image Registration

The quality of the stitched image mainly depends on the accuracy of the image input. The main problem is to find the deformation to find the corresponding position of the pattern or feature point in the image to be sewn from the reference image [9]. You can calculate the value of each parameter in the mathematical model according to the corresponding relationship between the template or image properties.

#### 2.1.3. Image Fusion

The image synthesis strategy must minimize the effects of residual distortion and brightness differences between images in the combined effect. Goals include designing stitching images, adjusting and blending brightness, defining overlapping areas, and eliminating seams, etc. [10, 11]. Although different image stitching algorithms are different, the implementation steps of the panorama will be different, but the general process includes the above steps.

### 2.2. Medical Image Enhancement Algorithm

#### 2.2.1. Sequence Image Registration

Inputs are two adjacent images that may have position offsets. The image is transformed by the image transformation coefficient generated by the optimizer, and then it is determined whether or not the two images are registered according to a certain similarity determination principle [12, 13]. Here, we choose the type of transformation between two adjacent slice images as rigid transformation. Rigid transformation can be used to model the offset between images by horizontal offset, vertical offset, and rotation angle:

(1) $$\begin{array}{c} \left(\begin{array}{c} x_{r}\\ y_{r}\\ 1 \end{array}\right)=\left(\begin{array}{ccc} \cos\;\theta & -\sin\;\theta & \Delta x\\ \sin\;\theta & \cos\;\theta & \Delta y\\ 0 & 0 & 1 \end{array}\right)\left(\begin{array}{c} x_{s}\\ y_{s}\\ 1 \end{array}\right), \end{array}$$

where (*x*_*r*_, *y*_*r*_) and (*x*_*s*_, *y*_*s*_) are two corresponding pixels. Δ*x* is the horizontal offset between the two images, Δ*y* is the vertical offset between the two images, and *θ* is the rotation angle between the two images.

#### 2.2.2. Extracting the Feature Points of the Image

Since the physical positions of two adjacent slice images are different, the morphology of the organs will also undergo some changes, so the feature points that can overcome the invariance of rotation and scaling between the images can meet the needs of sequence images. Certain points on the two images must have a corresponding relationship, and the corresponding points are related through a feature description, so that the goal of finding the corresponding points is achieved [14–16]. The steps of SIFT feature point extraction and matching are as follows:

(2) $$\begin{array}{c} G\left(x,y,\sigma \right)=\frac{1}{2\pi \sigma^{2}}e^{-\left({\left(x-m/2\right)}^{2}+{\left(y-n/2\right)}^{2}\right)/2\sigma^{2}}, \end{array}$$

where *m* and *n* are the size of the nucleus and (*x*, *y*) is the coordinate of the image pixel. The larger the *σ*, the more blurred the image will be. Then, use the Gaussian check of formula (2) to blur the image:

(3) $$\begin{array}{c} L\left(x,y,\sigma \right)=G\left(x,y,\sigma \right)*I\left(x,y\right). \end{array}$$

At the same time, we have to build a Gaussian pyramid model of the image. The specific operation is to perform a series of twice downsampling of the image to obtain a series of images of different sizes, from large to small, from bottom to top to build a pyramid model.

(4) $$\begin{array}{c} \frac{\partial G}{\partial \sigma }=\sigma \nabla^{2}G,\\ \sigma \nabla^{2}G=\frac{\partial G}{\partial \sigma }\approx \frac{G\left(x,y,k\sigma \right)}{k\sigma -\sigma }. \end{array}$$

So there is

(5) $$\begin{array}{c} G\left(x,y,k\sigma \right)-G\left(x,y,\sigma \right)\approx \left(k-1\right)\sigma^{2}\nabla^{2}G. \end{array}$$

Since *k* − 1 is just a constant value, which does not affect the position of the extreme point, a simpler Gaussian difference function can be used instead of the Gaussian Laplace function.

(6) $$\begin{array}{c} D\left(x,y,\sigma \right)=\left(G\left(x,y,k\sigma \right)-G\left(x,y,\sigma \right)\right)*I\left(x,y\right)=L\left(x,y,k\sigma \right)-L\left(x,y,\sigma \right), \end{array}$$

that is, two adjacent layers of Gaussian blurred images are used for difference to obtain a Gaussian difference image. It can be seen from this that, in order to obtain the extreme point detection of *S* scales, *S*+2 DOG images are required, so a total of *S*+3 Gaussian blur images of different scales are required [17, 18].

The parameters needed to detect the key points are as follows: the first is the size of the Gaussian kernel, which is the size of the blur scale; the second is the number of fuzzy layers, that is, the number of layers in a group *S*; and the third is the number of groups. The relationship between *O*, *S*, and *σ* is as follows:

(7) $$\begin{array}{c} \begin{array}{cc} \sigma \left(o,s\right)=\sigma_{0}2^{0+s/S} & o\in \left[0,\ldots ,O-1\right],\;s\in \left[0,\ldots ,S+2\right] \end{array}, \end{array}$$

where *σ*_0_ is the size of the initial Gaussian blur kernel.

(8) $$\begin{array}{c} \begin{array}{cc} \sigma \left(s\right)=\sigma_{0}2^{\left(s/S\right)} & s\in \left[0,\ldots ,S+2\right] \end{array}. \end{array}$$

The positions of the detected key points are all discrete, and the true feature points may be on sub-pixels [19]. Therefore, the three-dimensional (*x*, *y*, *σ*) quadratic function is used to fit the pixels as shown in equation (9).

(9) $$\begin{array}{c} D\left(X\right)=D+\frac{\partial D^{T}}{\partial X}X+\frac{1}{2}X^{T}\frac{\partial D^{2}}{\partial X^{2}}X. \end{array}$$

Among them, *X*=(*x*, *y*, *σ*)^*T*^, then derivation, and when the equation is equal to 0, it is the extreme point position.

Find the Hessian matrix at the key point; the principal curvature can be obtained by a Hessian matrix *H* with two rows and two columns:

(10) $$\begin{array}{c} H=\left[\begin{array}{cc} D_{xx} & D_{xy}\\ D_{yx} & D_{yy} \end{array}\right],\\ \begin{array}{cc} Tr\left(H\right)=a+\beta & Det\left(H\right)=a\beta . \end{array} \end{array}$$

The eigenvalues *a* and *β* of *H* represent the gradients in the *x* and *y* directions, and the principal curvature of *D* is proportional to the eigenvalue of *H*; then

(11) $$\begin{array}{c} \frac{Tr{\left(H\right)}^{2}}{Det\left(H\right)}=\frac{{\left(a+\beta \right)}^{2}}{a\beta }=\frac{{\left(r\beta +\beta \right)}^{2}}{r\beta^{2}}=\frac{{\left(r+1\right)}^{2}}{r}. \end{array}$$

When the key point is located at the edge, this will happen to the two eigenvalues.

(12) $$\begin{array}{c} \frac{Tr{\left(H\right)}^{2}}{Det\left(H\right)}<\frac{{\left(r+1\right)}^{2}}{r}. \end{array}$$

Through the above steps, we have obtained a more stable key point.

#### 2.2.3. Matching Feature Points and Eliminating False Matching Pairs

Since the distance between two adjacent sliced images is very small, there is no overall magnification for two adjacent sliced images. In other words, the distance between the two feature points of the image is above and above the first image. Since the distance of the second picture is approximately the same, define the distance ratio as shown in equation (13) [19, 20].

(13) $$\begin{array}{c} \text{ratio}=\bar{\frac{p_{i}p_{j}}{\bar{q_{i}q_{j}}}}. \end{array}$$

If the calculated distance ratio exceeds 1 ± *σ*, then the pair of matching points is a correct match. Otherwise, delete this pair of matching points.

#### 2.2.4. Calculating Rigid Registration Parameters

The reason for using the full search is because the amount of translation and rotation between the two slices is uncertain, and the offset may be large or small, so first use a large interval in a large range to determine a determine the rough range, and then search in small intervals with small intervals, and finally get the offset amount [20, 21]. So the distance to a point we need to minimize can be expressed as follows:

(14) $$\begin{array}{c} \left(\Delta x_{e},\Delta y_{e},\theta_{e}\right)=\arg\;\underset{\Omega =\left(\Delta x,\Delta y,\theta \right)}{\min}{\sum_{i=1}^{N}\left\|T_{\left(\Delta x,\Delta y,\theta \right)}\left(p_{i}\right)-q_{i}\right\|}_{2}. \end{array}$$

In the above formula, *T* represents the image transformation matrix including horizontal and vertical offset and rotation angle, *p*_*i*_ and *q*_*i*_ are the feature points corresponding to each other, and *N* is the number of feature point pairs [22, 23]. Therefore, the rigid registration parameters can be obtained by minimizing the distance of all feature points. Since each dimension of the offset vector calculated by this method is discrete, that is, it is an integer, but the offset vector may also be at the sub-pixel level, we calculate the offset vector obtained by equation (14). As a result, interpolation and fitting are performed to obtain a sub-pixel level offset vector.

#### 2.2.5. Registration Parameter Optimization

For medical images such as human heads, the shape of the head is not affected because the head has a very hard skull, but for the cells, the result is very soft, so its shape is in the production process; it is easy to be destroyed, so in the existing research field [24–26], the following relationship can be established:

(15) $$\begin{array}{c} v\left(x,y\right)\nabla I_{r}\left(x,y\right)=I_{s}\left(x,y\right)-I_{r}\left(x,y\right). \end{array}$$

In the above formula, *I*_*r*_ represents the gray value of the reference image, *I*_*s*_ represents the gray value of the offset image, ∇*I*_*r*_(*x*, *y*) represents the gradient of the gray value at the pixel (*x*, *y*) point, and *v*(*x*, *y*) is the offset vector we need to request. Then, write *v*(*x*, *y*) alone on the left side of the equation; then, the above equation becomes

(16) $$\begin{array}{c} v\left(x,y\right)=\frac{\left(I_{s}\left(x,y\right)-I_{r}\left(x,y\right)\right)\nabla I_{r}\left(x,y\right)}{{\left\|\nabla I_{r}\left(x,y\right)\right\|}^{2}}. \end{array}$$

Since there is a situation where the gradient size is close to 0 on some pixels, in this case, we add a term to the denominator to make the equation more stable, and the equation becomes

(17) $$\begin{array}{c} v\left(x,y\right)=\frac{\left(I_{s}\left(x,y\right)-I_{r}\left(x,y\right)\right)\nabla I_{r}\left(x,y\right)}{{\left\|\nabla I_{r}\left(x,y\right)\right\|}^{2}+{\left(I_{s}\left(x,y\right)-I_{r}\left(x,y\right)\right)}^{2}}. \end{array}$$

According to the characteristics of the above formula, we can make an analysis. If the coefficient is added to the two denominators, then the above formula becomes

(18) $$\begin{array}{c} v\left(x,y\right)=\frac{\left(I_{s}\left(x,y\right)-I_{r}\left(x,y\right)\right)\nabla I_{r}\left(x,y\right)}{{\left\|\nabla I_{r}\left(x,y\right)\right\|}^{2}+k{\left(I_{s}\left(x,y\right)-I_{r}\left(x,y\right)\right)}^{2}}. \end{array}$$

Because of $a{\left\|\nabla I_{r}\left(x,y\right)\right\|}^{2}+k{\left(I_{s}\left(x,y\right)-I_{r}\left(x,y\right)\right)}^{2}\geq \sqrt{ka}\left\|\nabla I_{r}\left(x,y\right)\right\|\left(I_{s}\left(x,y\right)-I_{r}\left(x,y\right)\right)$, *v*(*x*, *y*) is affected by *k* and *a*, which is $v\left(x,y\right)\leq 1/\sqrt{ka}$.

## 3. Experimental Design of the Effect of Nursing Intervention on Preventing Gastrointestinal Surgical Incision Infection

### 3.1. Test Subject

In this trial, 80 patients with gastrointestinal surgery admitted to a hospital from 2019 to 2020 were selected and randomly divided into two groups with 40 people in each group. The experimental group was treated with operating room nursing intervention combined with traditional treatment methods; in the control group, conventional care combined with traditional treatment methods was used for treatment. The general information of these 80 patients is shown in Table 1. Analyze the patient's depression, anxiety, and unhealthy mood, the quality of life after the operation, the incidence of incision infection, and wound healing.

Exclusion criteria were as follows: pregnant or breastfeeding women, patients with a history of treatment of other malignant tumors, patients with severe heart, liver, kidney, and other serious diseases, and patients with incomplete clinical data that affect the analysis of experimental results.

### 3.2. Experimental Method

Before and after the nursing intervention in the operating room, the patient's doctor, psychiatrist, and nurse jointly participated in the survey of the two groups. The Depression Self-Assessment Scale, Anxiety Self-Assessment Scale, and the Self-Assessment Scale for Recognition of Intraoperative Nursing Intervention assess a study subject's depression and anxiety and whether it is a nursing intervention in the operating room and compare and analyze the effectiveness of nursing interventions in the operating room. The survey tool used in the survey method is a questionnaire. The questionnaire adopts Likert's five-level evaluation method, and the score ranges from 1 to 5, which respectively represent the 5 indicators of completely disagree, disagree, neutral, agree, and completely agree.The higher the score, the more consistent the point of view.

### 3.3. Establishing Model Evaluation Index System

The evaluation index is a specific evaluation item that is determined according to the evaluation purpose and can reflect the basic characteristics of the evaluation target. Indicators are specific, and measurable, and are the observation points of your target. Clear conclusions can be drawn from the actual observation of the object. Typically, the metrics system includes three levels of metrics. This is the relationship between gradual decomposition and improvement. Among these, the first-stage evaluation index and the second-stage evaluation index are relatively abstract and cannot be used as direct evaluation criteria. The three-level assessment indicator should be specific, measurable, and action-oriented, and can be used as a direct basis for assessment.

### 3.4. Statistical Processing

Statistical analysis was carried out with SPSS 13.0 statistical software. The significance of the difference was tested by one-way analysis of variance, the difference between the two groups was tested by LSD-t, and the degree of infection of the surgical incision was tested by group *t*-test. *P* < 0.05 is considered to be significant and statistically significant.

## 4. Effect of Nursing Intervention on Preventing Gastrointestinal Surgical Incision Infection

### 4.1. Evaluation Index System Based on Index Reliability Testing

Here, we perform reliability analysis on all reliability indicators of each object, and the reliability indicators we choose for each object are slightly different. The results are shown in Table 2.

Figure 1 shows the patient's understanding of the nursing intervention in the operating room, the patient's negative emotional state, the patient's postoperative complications, and the patient's incision infection status. The impact of the data on this experiment is very good (*α* > 0.8); the data obtained from the patient's operation time and hospitalization time indicators have an acceptable impact on this experiment (*α* > 0.7), indicating that the nursing intervention in the operating room in this article is effective; the six indicators selected to prevent the effect of gastrointestinal surgical incision infection are reasonable, which provide a basis for subsequent experiments.

### 4.2. Based on Questionnaire Data

#### 4.2.1. Analysis of the Acceptance of Nursing Intervention in Operating Room between Two Groups of Patients

Here, we analyze the patient's acceptance of nursing intervention in the operating room and investigate the patient's acceptance of intervention before and after surgery. The results are shown in Table 3.

As can be seen from Figure 2, it can be seen that the patients in the control group did not receive nursing intervention in the operating room and did not actively learn about nursing intervention in the operating room after surgery. In the control group, there was little difference in perception of nursing intervention in the operating room before and after surgery. The difference was statistically significant (*P* < 0.05); the experimental group received treatment with an operating room nursing intervention combined with traditional treatment methods during surgery and had a clear understanding of the operating room nursing intervention. The experimental group clearly understood the operating room before and after surgery. The perception of nursing intervention was significantly improved, and the difference was statistically significant (*P* < 0.05).

#### 4.2.2. Comparison of the Unhealthy Emotional State of the Two Groups of Patients

Here is a comparative analysis of the postoperative negative mood of the patients, and the analysis of the improvement of the negative mood brought by the operating room nursing intervention methods compared with the traditional conventional nursing methods. The results are shown in Table 4.

It can be seen from Figure 3 that the control group has improved various bad moods after surgery, and the difference is statistically significant (*P* < 0.05), while the experimental group has improved in bad mood after nursing intervention in the operating room. The difference was statistically significant (*P* < 0.05). The emotional status of the two groups was compared before and after the operation. The results showed that the experimental group had a significant improvement in various negative emotions after the nursing intervention in the operating room, and there was a significant difference (*P* < 0.05).

### 4.3. Based on Test Data

#### 4.3.1. Analysis Based on the Levels of Various Indicators of the Two Groups of Patients

Here, we analyze the data of various indicators of patients and analyze the advantages of operating room nursing intervention methods compared with traditional conventional nursing methods during and after surgery. The results are shown in Table 5.

It can be seen from Figure 4 that the comparison of the operating time, first bowel time, and various levels of surgical indicators between the inpatient groups in the experimental group was lower than that of the control group. The difference was statistically significant (*P* < 0.05). This proves that nursing interventions in the operating room improve the patient's surgical index level compared to conventional nursing methods and promote the incision to heal as quickly as possible.

#### 4.3.2. Comparison of Postoperative Complications in the Two Groups

Here, we compare the postoperative complications of patients and analyze the advantages of operating room nursing intervention methods compared with traditional conventional nursing methods. The results are shown in Table 6.

It can be seen from Figure 5 that the incidence of gastrointestinal complications in the experimental group was reduced from 32.76% to 13.36% compared to the control group; metabolic complications in the experimental group were reduced from 19.88% to 9.36% compared to the control group; compared with the control group, the mechanical complications of the experimental group were reduced from 15.55% to 14.52%, and the reduction was not large; this proved that the operating room nursing intervention method has a lower probability of complications than the traditional conventional nursing method. The patient recovers faster.

#### 4.3.3. Comparison of the Two Groups of Patients in terms of Postoperative Wound Infection

Here is a comparison of patients with postoperative incision infections, and analysis of the advantages of operating room nursing intervention methods compared with traditional conventional nursing methods. The healing status is divided into three standards: Grade A, Grade B, and Grade C. Grade A: the incision has no adverse reactions and the healing is good; Grade B: the incision is healed poorly, with effusion, hematoma, etc.; Grade C: the incision is purulent, and the healing is not satisfactory. The results are shown in Table 7.

It can be seen from Figure 6 that the incision infection rate and wound healing of the two groups of patients are compared: the incision infection rate of the test group is lower than that of the control group, and the wound healing is significantly better than that of the control group. The difference is statistically significant (*P* < 0.05). It proves that this nursing model can effectively reduce the incidence of postoperative infections in patients, promote wound healing as soon as possible, help improve the prognosis of patients, and improve the quality of life of patients.

## 5. Conclusions

The control of postoperative incision infection should start from the source, block the source of bacteria and the way of bacterial transmission, visit the patient before the operation, grasp the patient's mental state and psychological concerns, and eliminate the burden through explanation of the surgical procedure and psychological counselling. Emotional fluctuations will have a great impact on the recovery of the patient's condition, and bad emotions should be avoided as much as possible, so as not to cause the body's immunity to decrease, thereby effectively reducing the incidence of incision infection. Secondly, it is necessary to ensure a sterile and clean operating room environment, which requires a certain time interval between the two operations. Medical staff should strengthen hand cleaning, change surgical gloves after exploring the body cavity, and apply a skin protective film to the patient's incision site. Cover with a clean bag to protect the incision from infection. In this article, patients in the experimental group received nursing intervention in the operating room. Analysis of the results found that the postoperative rehabilitation indicators of the experimental group were better than those of the control group. The excellent incision healing rate reached 92.5% and the incision infection incidence rate was 5%, which was lower than that of the control group, which reflects the effectiveness of the care model. Nursing intervention in the operating room reduces the infection rate at the patient's incision site, improves the patient's level of surgical indicators, and promotes healing of the incision site as soon as possible, greatly improving the safety of clinical treatment, and is of more value. The downside of this study is that, at the design stage of the study, it was not taken into account that the genders of patients may have different psychological endurances and that they may have certain effects on the outcome of psychological interventions and should be considered.

## Figures and Tables

**Figure 1:** Indicator reliability test analysis chart.

**Figure 2:** Analysis chart of patients' acceptance of nursing intervention in operating room.

**Figure 3:** Analysis chart of patient's unhealthy emotional state.

**Figure 4:** Analysis chart of the levels of various indicators in the two groups.

**Figure 5:** Analysis of the patient's postoperative complications.

**Figure 6:** Analysis diagram of patients with postoperative wound infection.

**Table 1:** General information of the two groups of patients.

Group	Number of cases		Years	Course of disease	Years of education
	Male	Female			
Experiment group	24	16	56.72 ± 6.21	84 ± 5.5	11 ± 3.12
Control group	22	28	56.98 ± 6.02	84 ± 3.4	11 ± 2.57

**Table 2:** Data sheet of evaluation index system for index reliability testing.

	Very clear	Clear	General	Not clear	Chaotic	Alpha
Operation time	3.85	3.61	4.21	0.54	0.49	0.7216
Hospital stay	3.96	4.18	3.84	0.47	0.38	0.7533
Understanding of nursing intervention	3.91	4.14	4.01	0.56	0.38	0.8417
Bad mood	3.69	4.24	3.97	0.68	0.57	0.8692
Complication	3.69	4.14	4.08	0.52	0.55	0.8273
Incision infection	3.60	3.83	4.74	0.41	0.46	0.8337

**Table 3:** Patient's acceptance score sheet for nursing intervention in operating room.

Score	1	2	3	4	5
Experiment group before surgery	2.83	3.10	2.98	2.73	2.73
Experiment group after surgery	4.83	4.87	4.42	4.98	4.38
Control group before surgery	3.04	3.31	3.30	3.39	3.56
Control group after surgery	2.78	3.42	3.10	2.71	3.53
*t*	6.523	4.256	7.331	6.289	5.982
*P*	<0.001	<0.001	<0.001	<0.001	<0.001

**Table 4:** Patient's bad emotional state data sheet.

Attribute	Fear	Anxiety	Depression	Tension	Worry
Experiment group before surgery	2.59	2.48	2.61	2.46	2.62
Experiment group after surgery	2.02	2.18	2.07	1.95	1.95
Control group before surgery	2.49	2.40	2.51	2.33	2.76
Control group after surgery	4.38	4.28	4.08	4.06	4.22
*t*	11.326	7.654	7.233	7.472	8.175
*P*	0.012	0.010	0.009	0.005	0.008

**Table 5:** Data table of various index levels.

Group	Operation time (min)	First exhaust time (d)	Time to first bowel movement (d)	Hospital stay (d)
Experiment group	60.85	1.47	1.21	10.65
Control group	90.87	3.54	3.41	16.95
*t*	3.478	5.542	2.360	6.244
*P*	0.001	0.001	0.001	0.001

**Table 6:** Data sheet of the patient's postoperative complications.

Complication	Experiment group		Control group		*t*	*P*
	Probability	Rank	Probability	Rank		
Vomiting	12.36	56.58	32.76	50.59	2.813	0.027
Bloating	11.72	57.61	31.74	50.72	2.270	0.021
Diarrhea	10.63	54.32	27.55	53.27	2.012	0.032
High blood sugar	9.36	57.09	19.88	50.63	1.098	0.012
Hypoglycemia	8.98	57.89	19.13	53.14	2.453	0.025
Blocking the pipe	14.52	57.32	15.55	50.71	3.447	0.329

**Table 7:** Data sheet for patients with postoperative wound infection.

Group	Incision healing			Incision infection rate
	Grade A	Grade B	Grade C	
Experiment group	20 (50%)	17 (42.5%)	1 (2.5%)	2 (5%)
Control group	15 (37.5%)	10 (25%)	5 (12.5%)	10 (25%)
*T*	1.749	4.832	7.246	6.600
*P*	0.216	0.455	0.009	0.012

## Data Availability

Data sharing is not applicable to this article as no datasets were generated or analyzed during the current study.
